# Factors Related to Depression and Mental Health That Affect the Quality of Life of the Elderly

**DOI:** 10.1155/2022/7764745

**Published:** 2022-11-16

**Authors:** Ji Eun Park, Ryoung Choi

**Affiliations:** ^1^Department of Nursing, Keimyung College University, Daegu, Republic of Korea; ^2^Department of Health Administration, Dongshin University, Naju, Republic of Korea

## Abstract

The purpose of this study was to provide basic data for the healthcare of the elderly by identifying the effects of depression and quality of sleep on the lives of the elderly. The subjects of this study were 120 elderly people who used the elderly welfare center and senior citizen center in one of the cities in South Korea, who understood the purpose of the study and signed the consent form for participation in the study. This study is a descriptive correlation study using a questionnaire to compare and analyze the effects of depression and quality of sleep on the quality of life of the elderly. Data were analyzed using the SPSS 25.0 program. According to general characteristics, the level of depression, quality of sleep, and quality of life were analyzed by frequency, percentage, mean, and standard deviation. The level of depression, quality of sleep, and quality of life, as measured by the general characteristics, were evaluated by the *t*-test and ANOVA. The quality of life, depression, and quality of sleep were analyzed by Pearson's correlation analysis. Linear regression analysis was performed to analyze the factors influencing sleep quality. As a result of this research, depression, psychological, and social domains had positive correlations, and depression and biological domains had negative correlations. As a result of this research, quality of sleep was found to have a negative correlation with the psychological domain and quality of sleep was found to have a positive correlation with the biological environment domain. Based on this research, this author proposes that research should be attempted later with the elderly who were classified as the elderly who are living alone, the elderly who are living at home, and the elderly at the facilities as the subjects. Therefore, depression and the quality of sleep have a big influence on the health condition of the elderly because they may be the important health problems that cannot be overlooked in terms of the quality of life. Furthermore, there is a need to develop a continuous, specific, and practical healthcare program that can manage depression and quality of sleep in old age.

## 1. Introduction

With the industrialization of modern society in the 21st century due to the development of medicine and science, the quality of life has been increasing. In addition, with the improvement in the quality of medical treatment, the elderly population has also been increasing rapidly. Among the total population as of 2019, the elderly who are 65 years old and older accounted for 14.9%, which means that they have already entered the elderly society. Moreover, it is anticipated that, until the year 2067, it will increase by 46.5% [1].

Although depression can appear throughout the whole process of the developmental phases of human beings, it has received attention because it is a psychological and social characteristic of the elderly [2].

Regarding the depression of the elderly, the lowering of the ability to adapt to the many changes appears by generally experiencing the internal and external changes caused by aging from a psychological aspect. At this time, the psychological change that stands out is the anxiety or feeling of depression due to stress. Then, this acts as a cause that lowers not only the level of satisfaction regarding life but also the quality of life [3]. To the elderly, depression is a cause that lowers self-esteem and quality of life [4–6]. In addition, it also has a negative influence on the quality of life of the elderly in the social and national dimensions by causing problems such as functional disorders in everyday life activities, sleep disorders, and suicide acts due to important health problems, so health management of the elderly is needed [7, 8].

The elderly cannot have deep sleep at night as the amplitude of the circadian rhythm is decreased by a change in the biorhythm. Therefore, they wake up frequently or show the phenomenon of daytime sleepiness. In addition, with the changes in sleep patterns, their sleep latency continues and their sleep efficiency decreases. According to a recent investigation into the health and nutrition of the citizens, in South Korea, the elderly, whose average sleep time was less than 6 hours, accounted for 27% [9]. In order to live a healthy aged life, the quality of sleep of the elderly is important. The quality of sleep varies from individual to individual. The quality of sleep also becomes different with age. As for the characteristics of the sleep of the elderly, although there is no change in the entire sleep time, low-quality sleep can exist [10]. In other words, it takes a long time until falling asleep. In addition, they wake up frequently while sleeping. Once they wake up, they find it difficult to fall asleep again. Sleep problems are common among the elderly [11].

Quality of life may be a multidimensional concept that means the subjective sense of satisfaction that each and every individual feels under objective conditions, which means the condition of the well-being physically and mentally [12]. In old age, the quality of life gets lowered in all of the physical, functional, mental, and social domains due to the weakening of the physical functions related to aging and facing a psychological, social, or economic crisis situation [11]. Especially, the depression that appears among the elderly gets connected to the loss of the role and the dependent life [13]. Old age may be a time when there is more role loss than at any other phase in the development of life. During the time of such a loss, the elderly can easily fall into a state of depression. In addition, the worsening of health, bereavement, and economic difficulty can also lower the overall quality of life of the elderly. As for the approach to solving the problem of the mental health of the elderly, a general approach is needed in the social, economic, and psychological aspects.

In order to be able to live a healthy and happy aged life, efforts for understanding and supporting are continuously needed [14, 15]. As the quality of sleep is influenced by a psychological aspect such as depression, depression is an important health problem that lowers the quality of sleep.

Depression and the quality of sleep have a big influence on the health condition of the elderly because they may be important health problems that cannot be overlooked in terms of the quality of life. Therefore, the purpose of this study is to provide basic data for the healthcare of the elderly by investigating the effects of depression and quality of sleep on the lives of the elderly.

## 2. Methods

### 2.1. Respondents of the Study

The respondents of this study were 120 elderly people who used the elderly welfare center and senior citizen center in one of the cities in South Korea, who understood the purpose of the study and signed the consent form for participation in the study.

### 2.2. Research Instruments

#### 2.2.1. Depression

The Geriatric Depression Scale Short Form-Korea Version, GDSSF-K, which Ki had translated and standardized from the GDS Short Form, which was developed by Sheikh and Yesavege, had been used [16], and with a total of 15 questions, in the case of “Yes,” it was 1 point. In the case of “No,” it was 0 point. The higher the score, the greater the extent of the depression. Also, according to the score, 0 point to 4 points is classified as normal, 5 points to 9 points is classified as slight depression, and 10 points to 15 points is classified as serious depression. Among the total of 15 questions, 10 questions were positive questions, and regarding these positive questions, they were reverse converted. The higher the score, the greater the extent of the depression.

At the time of development, the reliability was Cronbach's *α* = .94. In this study, the reliability was Cronbach's *α* = .90.

#### 2.2.2. Quality of Sleep

In order to measure the quality of sleep, a tool developed by Kwon has been used [17]. Regarding the tool for measuring the quality of sleep, there had been 15 questions. Regarding each question, with the Likert scale of 5 points, it had been organized with the scale from 1 point for “Not at all so” to 5 points for “It is always so.” Also, the higher the score, the worse the quality of sleep.

At the time of development, the reliability was Cronbach's *α* = .89. In this study, the reliability was Cronbach's *α* = .94.

#### 2.2.3. Quality of Life

In order to measure the quality of life, the Korean version of the WHOQOL-BREF [18] that had been revised based on the WHOQOL-100, which was developed by the WHO, had been used. Also, regarding this research, with the 8 questions in the domain of physical health, the 6 questions in the psychological domain, the 2 questions in the social domain, and the 8 questions in the living environment domain, it is organized with a total of 24 questions in the 4 domains. The measurement of each question had been a 5 points scale from “Not at all so” 1 point to “Very much so” 5 points. Also, the higher the score, the better the quality of life

At the time of development, the reliability was Cronbach's *α* = .89. In this study, the reliability was Cronbach's *α* = .90.

### 2.3. Data Analysis

The data of this study were analyzed by using SPSS (ver. 25.0). The general characteristics such as the level of depression, quality of sleep, and quality of life were analyzed by frequency, percentage, mean, and standard deviation. The levels of depression, quality of sleep, and quality of life as measured by the general characteristics were evaluated by *t*-test and ANOVA. The quality of life, depression, and quality of sleep were analyzed by Pearson's correlation analysis. A linear regression analysis was performed to analyze the factors influencing sleep quality.

## 3. Results

### 3.1. General Characteristics of Subjects

Regarding the gender, it appeared that the males were 18.3% and the females were 81.7%. The average age was 74.98 years old. Regarding the academic background, the junior high school graduates or lower were the majority at 73.3%. Regarding religion, Buddhism was the most at 45.0%. The housemate is the spouse, with the most at 50.8%. The average number of children was 2.78 persons. Regarding whether or not there are children to rely on, it appeared that “There are” was 90.8% and “There are not” was 9.2%. Regarding the person who gives help and pays attention at ordinary times, the children were the most at 50.0%. Regarding the number of times the gathering occurred, 1 time or more in two months was the most at 43.3%. Regarding whether or not there is a workplace, it appeared as “There is not” at 87.5% and “There is” at 12.5%. Regarding the economic level, ordinary was the most at 68.3%, and it appeared in the order of being on the difficult side at 16.7% and on the side of living well at 15%. Regarding the allowance for one month, 300,000 won or less was the most at 32.5%. Regarding the subjective condition of the population's health, ordinary was the most at 46.7%. Also, it appeared in the order of being on the side of being bad at 23.3%, on the side of being good at 21.7%, on the side of being very bad at 4.2%, and on the side of being very good at 4.2%. Regarding whether or not there is an illness, it appeared that “There is” was 67.5% and “There is not” was 32.5% (Table 1).

### 3.2. Degree of Depression

As for the degree of depression, the mean of the total score was 3.67. For the question about depression, “Do you frequently feel unrest regarding trivial affairs?” The score was 0.39, “Are you hopeful regarding the future?” The highest score was 0.39. On the other hand, “Do you feel that you are happy during most of the time?” scored 0.15, and “Is your mind comfortable like before?” The lowest score was 0.15 points (Table 2).

### 3.3. Quality of Sleep

As for the quality of sleep, the average of the total score was 3.85. As for the quality of sleep, “If I wake up while sleeping at night, it is difficult for me to fall asleep again” had the highest score, with 2.53 points, and “I cannot sleep deeply at night” had 2.43 points. The score of 2.34 for “I cannot fall asleep well even when I am lying down in order to sleep at night” and 2.34 for “Although the time of lying down on the bed is long, the time of actually sleeping is short” was found with a score of 2.34. “Sometimes, I wake up because my legs suddenly tremble or flinch while sleeping” was the lowest at 1.60 points (Table 3).

### 3.4. Quality of Life

As for the quality of life, the average of the total score was 3.54. In all domains, the living environment area had the highest average score of 3.70 points, the psychological domain averaged 3.60 points, the social domain 3.45 points, and the physical domain 3.42 points. In the physical domain, “Satisfied with my capability to carry on with my everyday life” showed the highest score of 3.68. The lowest score of 3.04 was “A lot of the medical treatment is needed for me to do well in my everyday life.” In the psychological realm, “It is not a negative mood, including being depressed, the feeling of despair, the anxiety, the low-spiritedness, etc.” It was the highest with 3.81 points. “I accept my physical appearance” was the lowest with 3.39 points. In the social domain, “Satisfied with the help of my friend” showed 3.50 points. “I evaluate the quality of my life as being good” showed 3.49 points. In the living environment area, “I have been living in a residential environment, which is good for health,” showed the highest score of 3.93. “I have sufficient money that is needed” showed the lowest score of 3.09 (Table 4).

### 3.5. Depression according to General Characteristics

In the verification of the difference in the degree of depression according to general characteristics, “none” showed the highest score of 4.32 in relation to the number of meeting participations. “Once every 2 weeks” showed the highest score with an average of 4.00, “once a month” with an average of 4.00, and “once a week” with an average of 2.80 points. They showed a statistically significant difference (*p* = 0.024). As for the economic level, “economic hardship” was the highest with 5.90 points. “Being ordinary” scored 3.32 points and “pretty rich” scored 2.77 points. There was a statistically significant difference (*p* = 0.003). As for the average monthly allowance, “100,000 won or less” showed the highest score with 4.38 points, “300,000 won or less” with 4.02 points, “200,000 won or less” with 4.00 points, and “400,000 won or less” with 3.83 points, “500,000 won or less” with 2.50 points. They showed a statistically significant difference (*p* = 0.044). As for the subjective status of health, “very bad” was the highest with 9.20 points, “Ordinary” was 5.10 points, “normal” was 3.10 points, “good” was 2.80 points, and “very good” was 1.0 points in that order. This showed a statistically significant difference (*p* = 0.001) (Table 5).

### 3.6. Quality of Sleep according to General Characteristics

Regarding the verification of the difference in the extent of the sleep resulting from the general characteristic in relation to the question of, “Do you have children who can be relied on?” “Yes” was 3.99 points and “No” was 3.44 points. These showed statistically significant differences (*p*=0.034). As for the economic level, “high” showed the highest score of 4.08, followed by “medium” at 4.04 and “low” at 3.51. There was a statistically significant difference (*p*=0.005). As for the subjective state of health, “very healthy” showed the highest score with 4.54 points, followed by “healthy” with 4.22 points, “ordinary” with 3.93 points, “very unhealthy” with 3.76 points, and “unhealthy” with 3.49 points. They showed a statistically significant difference (*p*=0.001) (Table 6).

### 3.7. Quality of Life according to General Characteristics

Regarding the verification of the difference in the extent of the quality of life resulting from the general characteristic, in relation to gender, “female” was 87.11 points and “male” was 80.31 points. These showed statistically significant differences (*p*=0.005). As for the number of children, “5 persons or more” had the highest score with 91.8 points, “3 persons or more” with 88.72 points, “2 persons or more” with 83.06 points, and “1 person or fewer” with 91.8 points and 65.45 points. There was a statistically significant difference (*p*=0.010). As for participation recruitment, “the elderly volunteer service organization” showed the highest score of 101.0, followed by “the senior college” with 88.33 points, “the senior citizens” “center” with 88.04 points, and “none” with 82.40 points. They showed a statistically significant difference (*p*=0.041). As for the number of meetings, “more than once a week” showed the highest score at 90.97, “more than once every 2 weeks” at 80.85 points, “more than once a month” at 86.64 points, and “more than once every 2 months” at 80.85 points and 81.71 points. There was a statistically significant difference (*p*=0.003). As for the economic level, “pretty rich” showed the highest score at 97.55, followed by “ordinary” at 85.32 and “economic hardship” at 77.55. They showed a statistically significant difference (*p*=0.001). As for the monthly allowance, “500,000 won or more” showed the highest score at 91.13 points, “200,000 won or less” 87.08 points, “500,000 won or less” at 86.66 points, “300,000 won or less” at 83.2 points, and “100,000 won or less” appeared in order with 82.04 points. There was a statistically significant difference (*p*=0.033). As for the subjective state of health, “very good” scored the highest with 110.8 points, followed by “good” with 91.46 points, “ordinary” with 84.53 points, “bad” with 82.60 points, and “very bad” with 65.0 points. This showed a statistically significant difference (*p*=0.001) (Table 7).

### 3.8. Correlation between Depression Level, Quality of Sleep, and Quality of Life

Depression and psychological domains have a positive correlation (*r* = −0.270, *p*=0.003). There is a positive correlation between depression and social domains (*r* = 0.245, *p*=0.007). There is a negative correlation between depression and the biological domain (*r* = −0.205, *p*=0.024). Sleep quality has a negative correlation with the psychological domain (*r* = −0.455, *p*=0.001). Sleep quality has a positive correlation with the biological environment (*r* = 0.419, *p*=0.001) (Table 8).

### 3.9. Factors Affecting the Quality of Life

In the physical domain, the higher the number of children, the lower the quality of life (*β* = 0.302, *p*=0.010). In the psychological domain, the quality of life deteriorated when there was a job (*β* = −0.287, *p*=0.002). The higher the quality of sleep, the lower the quality of life (*β* = −0.348, *p*=0.001). In the social domain, the higher the economic level, the lower the quality of life *(β* = −0.288, *p*=0.004). The quality of life decreases as the health status increases *(β* = 0.280, *p*=0.018). In the living-environment domain, the quality of life decreases with disease (*β* = −0.216, *p*=0.025). The worse the quality of sleep, the lower the quality of life (*β* = 0.436, *p*=0.001) (Table 9).

## 4. Conclusions

The purpose of this study was to provide basic data for the healthcare of the elderly by identifying the effects of depression and quality of sleep on the lives of the elderly.

The summarized conclusions of this research are as follows: the extent of the depression in the subjects was low, with an average total score of 3.67 points; the quality of sleep was low with an average of 3.85 points; and the quality of life had an average of 85.86 points, which was low the medium level.

The difference in the degree of depression according to the general characteristics was higher as the number of meeting participants decreased, the financial difficulties increased, the average monthly allowance decreased, and the health status was poor with the depression elderly experienced. As for the difference in sleep quality according to general characteristics, the more children you can depend on, the better the economic level, and the better the health, the better the sleep quality.

As for the difference in the quality of life according to general characteristics, the more children, the more people participating in the elderly volunteer group, the more frequent the meetings, the higher the standard of living, and the higher the allowance for one month. Also, the quality of life of women was higher than that of men.

As a result of this research, differences in depression, sleep, and quality of life among the elderly according to general characteristics were identified. Depression, psychological, and social domains had positive correlations, and depression and biological domains had negative correlations.

Sleep quality was found to have a negative correlation with the psychological domain, and sleep quality was found to have a positive correlation with the biological environment domain. Based on this research, this author proposes that research should be attempted later with the elderly who were classified as the elderly who are living alone, the elderly who are living at home, and the elderly at the facilities as the subjects. In addition, there is a need to develop a continuous, specific, and practical intervention program that can manage depression and sleep quality in old age.

## Figures and Tables

**Table 1:** General characteristics.

Characteristics	Categories	*n*	%
Gender	Male	22	18.3
	Female	98	81.7

Age (year)	65–69	34	28.3
	70–79	58	48.4
	≥80	28	22.4

Religion	Buddhism	54	45.0
	Christianity	14	11.7
	Catholic	17	14.2
	No religion	35	29.2

Education	Junior high school graduate	88	73.3
	High school graduate	24	20.0
	University graduate or higher	8	6.7

Marital status	Married	67	55.8
	Bereavement, separation, divorce	52	43.3
	Single	1	0.8

Living together	Couple	61	50.8
	Married children	21	17.5
	Unmarried children	7	5.8
	Alone	31	25.8

Number of children	0–1	11	9.1
	2	47	39.2
	3–4	51	42.5
	≥5	11	9.2

Dependent child	Has	109	90.8
	None	11	9.2

A person who usually cares and helps	Marriage partner	42	35.0
	Children	60	50.0
	Neighbors and others	18	15.0

Meeting	Senior citizen's center	48	40.0
	Senior college	15	12.5
	Senior volunteer group	3	2.5
	None	54	45.0

Number of meetings	Once a week	47	39.2
	Once in two weeks	7	5.8
	Once a month	14	11.7
	Once in two months	52	43.3

Occupation status	Has	15	12.5
	None	105	87.5

Economic level	Low	20	16.7
	Medium	82	68.3
	High	18	15.0

Monthly allowance	≥100,000 won	21	17.5
	≥200,000 won	12	10.0
	≥300,000 won	39	32.5
	≥400,000 won	18	15.0
	≥500,000 won	30	25.0

Subjective health status	Very healthy	5	4.2
	Healthy	26	21.7
	Average	56	46.7
	Unhealthy	28	23.3
	Very unhealthy	5	4.2

Disease status	Has	81	67.5
	None	39	32.5

**Table 2:** Degree of depression.

Domain	Classification	Mean (SD)
Degree of depression	(1) Are you satisfied with your usual life?	0.15 (1.35)
	(2) Have you had a lot of diminished activity and interest?	0.30 (0.46)
	(3) Are you hopeful for the future?	0.39 (0.49)
	(4) Do you spend most of your time in a clear mind?	0.06 (0.25)
	(5) Do you feel happy most of the time?	0.15 (0.36)
	(6) Do you think it is beautiful to be alive now?	0.17 (0.38)
	(7) Do you sometimes feel discouraged and depressed?	0.33 (0.47)
	(8) Do you feel that your life is not very worthwhile now?	0.20 (0.40)
	(9) Do you find life very interesting?	0.27 (0.44)
	(10) Do you feel full of vitality?	0.21 (0.41)
	(11) Do you often feel agitated by the little things?	0.39 (0.49)
	(12) Do you often feel like you want to cry?	0.22 (0.41)
	(13) Do you enjoy waking up in the morning?	0.25 (0.43)
	(14) Are you easy to make decisions?	0.35 (0.48)
	(15) Is your mind as comfortable as before?	0.15 (0.36)
Total score average		3.67 (3.33)

**Table 3:** Quality of sleep.

Domain	Classification	Mean (SD)
Quality of sleep	(1) I can't sleep well even when I lay down to sleep at night	2.34 (1.22)
	(2) It is difficult to fall asleep again after waking up after sleeping at night	2.53 (1.25)
	(3) I can't sleep deeply at night	2.43 (1.25)
	(4) When I wake up at dawn, I can't sleep until morning even if I want to sleep more	2.33 (1.21)
	(5) Even after sleeping, I wake up frequently because of aches or pains	1.80 (1.17)
	(6) When I lie down to sleep, I can't sleep because of a tingling, aching, or tingling feeling in my legs	1.76 (1.12)
	(7) I sometimes wake up because my legs tremble or flutter while I'm sleeping	1.60 (1.05)
	(8) I barely wake up in the morning	1.62 (1.06)
	(9) It takes a lot of time to get out of bed	1.75 (1.16)
	(10) I am constantly tired during the day because I can't sleep well	2.20 (1.25)
	(11) I keep getting sleepy even after I wake up in the morning	1.88 (1.20)
	(12) My body is heavy because I can't sleep well	1.97 (1.18)
	(13) I think I can't sleep well	2.20 (1.25)
	(14) I feel lack of sleep	2.04 (1.20)
	(15) The time to lie in bed is long, but the time to actually sleep is short	2.34 (1.36)
Total score average		3.85 (0.75)

**Table 4:** Quality of life.

Domain	Classification	Mean (SD)
Physical domain	(1) Satisfied with my health	3.21 (1.10)
	(2) You need a lot of treatment to do your daily life well	3.04 (1.08)
	(3) Physical pain hinders work	3.36 (1.22)
	(4) You have enough energy to do your daily life	3.54 (0.96)
	(5) I can get around well	3.60 (1.07)
	(6) Satisfied with sleep	3.57 (1.00)
	(7) Satisfied with my ability to perform daily life	3.68 (1.02)
	(8) Satisfied with my ability to work	3.55 (1.03)
Total score average		3.42 (0.21)

Psychological domain	(1) Enjoy life	3.63 (0.21)
	(2) I feel that my life is somewhat meaningful	3.61 (0.91)
	(3) I can concentrate my mind well	3.61 (1.00)
	(4)I agree with my physical appearance	3.39 (0.97)
	(5) Satisfied with myself	3.56 (1.04)
	(6) Not a negative mood, such as depression, feelings of restlessness, anxiety, or depression	3.81 (1.22)
Total score average		3.60 (0.13)

Social domain	(1) I appreciate the quality of my life	3.49 (0.88)
	(2) Satisfied with the help of a friend	3.50 (1.02)
Total score average		3.45 (0.08)

Living environment domain	(1) Feeling safe in everyday life	3.69 (0.95)
	(2) I live in a healthy living environment	3.93 (0.82)
	(3) You have enough money for what you need	3.09 (1.00)
	(4) You can easily get the information you need for your daily life	3.45 (1.00)
	(5) Have an opportunity to enjoy leisure	3.86 (0.81)
	(6) Satisfied with the easy access to medical services	3.87 (0.86)
	(7) I am satisfied with the house I live in and the conversion landscape	3.84 (0.87)
	(8).Satisfied with the mode of transportation I use	3.89 (0.84)
Total score average		3.70 (0.29)
Total question average		3.70 (0.29)

**Table 5:** Depression according to general characteristics.

Variable	Classification	Mean (SD)	*t*	*p*
Gender	Male	4.45 (3.82)	1.47	0.226
	Female	3.50 (3.20)		

Age (year)	65–69	3.05 (2.67)	0.883	0.452
	70–79	3.67 (3.53)		
	≥80	4.69 (3.27)		

Religion	Buddhism	3.55 (3.05)	0.940	0.749
	Christianity	4.35 (3.45)		
	Catholic	4.58 (3.72)		
	No religion	3.14(3.50)		

Education	Junior high school graduate	3.73 (3.51)	0.178	0.615
	High school graduate	3.66 (2.98)		
	University graduate or higher	3.00 (2.32)		

Marital status	Married	3.35 (2.89)	2.344	0.143
	Bereavement, separation, divorce	3.96 (3.75)		
	Single	1.00 (1.00)		

Living together	Couple	3.34 (2.93)	0.415	0.304
	Married children	3.95 (3.41)		
	Unmarried children	3.85 (2.91)		
	Alone	4.09 (4.10)		

Number of children	0-1	3.70 (4.37)	1.149	0.239
	2	3.87 (3.23)		
	3-4	3.61 (3.23)		
	≥5	2.64 (1.39)		

Dependent child	Has	3.49(3.15)	3.524	0.063
	None	5.45(4.56)		

A person who usually cares and helps	Marriage partner	3.26(3.26)	0.950	0.755
	Children	4.08(3.48)		
	Neighbors and others	2.96(1.87)		

Meeting	Senior citizen's center	3.16(2.77)	1.328	0.145
	Senior college	3.93(3.88)		
	Senior volunteer group	1.33(0.57)		
	None	4.18(3.64)		

Number of meetings	Once a week	2.80(2.87)	1.825	0.024
	Once in two weeks	4.00(2.16)		
	Once a month	4.00(3.72)		
	Once in two months	4.32(3.63)		

Occupation status	Has	3.53(3.13)	0.031	0.861
	None	3.69(3.37)		

Economic level	Low	2.77(3.22)	6.016	0.003
	Medium	3.32(2.88)		
	High	5.90(4.29)		

Monthly allowance	≥100,000 won	4.38(3.36)	1.328	0.044
	≥200,000 won	4.00(3.04)		
	≥300,000 won	4.02(4.05)		
	≥400,000 won	3.83(3.34)		
	≥500,000 won	2.50(2.02)		

Subjective health status	Very healthy	9.20(3.27)	7.844	0.001
	Healthy	5.10(3.98)		
	Average	3.10(2.55)		
	Unhealthy	2.80(2.85)		
	Very unhealthy	1.00(1.00)		

Disease status	Has	3.83(3.55)	0.207	0.438
	None	3.33(2.82)		

**Table 6:** Quality of sleep according to general characteristics.

Variable	Classification	Mean (SD)	*t*	*p*
Gender	Male	3.81 (0.83)	0.458	0.513
	Female	3.92 (0.75)		

Age (year)	65–69	4.17 (0.12)	1.197	0.889
	70–79	3.79 (0.10)		
	≥80	4.25 (0.27)		

Religion	Buddhism	3.90 (0.78)	1.694	0.352
	Christianity	3.55 (0.72)		
	Catholic	3.85 (0.75)		
	No religion	4.12 (0.77)		

Education	Junior high school graduate	3.95 (0.80)	0.006	0.951
	High school graduate	3.94 (0.79)		
	University graduate or higher	3.95 (0.76)		

Marital status	Married	3.97 (0.75)	0.839	0.590
	Bereavement, separation, divorce	3.84 (0.79)		
	Single	4.68 (0.00)		

Living together	Couple	3.98 (0.71)	0.496	0.778
	Married children	3.78 (0.85)		
	Unmarried children	3.72 (1.08)		
	Alone	3.95 (0.75)		

Number of children	0-1	3.57 (0.91)	1.705	0.356
	2	4.06 (0.73)		
	3-4	3.92 (0.70)		
	≥5	4.06 (0.82)		

Dependent child	Has	3.99 (0.73)	4.359	0.034
	None	3.44 (0.95)		

A person who usually cares and helps	Marriage partner	3.91 (0.75)	1.067	0.435
	Children	3.99 (0.79)		
	Neighbors and others	3.83 (0.77)		

Meeting	Senior citizen's center	3.90 (0.75)	0.443	0.729
	Senior college	3.89 (0.84)		
	Senior volunteer group	4.39(0.32)		
	None	3.92 (0.79)		

Number of meetings	Once a week	4.15 (0.81)	2.423	0.162
	Once in two weeks	3.45 (0.39)		
	Once a month	3.72 (0.61)		
	Once in two months	3.85 (0.75)		

Occupation status	Has	4.10 (0.70)	0.382	0.435
	None	3.91 (0.79)		

Economic level	Low	3.51(0.75)	5.788	0.005
	Medium	4.04 (0.74)		
	High	4.08 (0.76)		

Monthly allowance	≥100,000 won	3.78 (0.78)	0.436	0.540
	≥200,000 won	3.91 (0.84)		
	≥300,000 won	3.85 (0.72)		
	≥400,000 won	4.16(0.69)		
	≥500,000 won	3.94 (0.78)		

Subjective health status	Very healthy	4.54 (0.42)	4.536	0.001
	Healthy	4.22 (0.70)		
	Average	3.93 (0.75)		
	Unhealthy	3.49 (0.78)		
	Very unhealthy	3.76 (0.68)		

Disease status	Has	3.95 (0.80)	0.021	0.886
	None	3.92 (0.76)		

**Table 7:** Quality of life according to general characteristics.

Variable	Classification	Mean (SD)	*t*	*p*
Gender	Male	80.31 (14.04)	3.882	0.05
	Female	87.11 (14.73)		

Age (year)	65–69	88.73 (16.84)	0.661	0.671
	70–79	84.67 (13.96)		
	≥80	87.00 (15.01)		

Religion	Buddhism	86.12 (14.39)	2.673	0.275
	Christianity	78.21 (16.67)		
	Catholic	82.41 (16.28)		
	No religion	90.20 (12.73)		

Education	Junior high school graduate	86.34 (14.71)	1.676	0.915
	High school graduate	81.95 (15.21)		
	University graduate or higher	92.37 (12.85)		

Marital status	Married	87.82 (14.16)	2.065	0.070
	Bereavement, separation, divorce	83.73 (15.28)		
	Single	66.00 (0.00)		

Living together	Couple	87.95 (14.41)	0.970	0.091
	Married children	85.38 (11.10)		
	Unmarried children	83.71 (13.97)		
	Alone	82.58 (17.60)		

Number of children	0-1	65.45 (16.38)	2.082	0.010
	2	83.06 (15.49)		
	3-4	88.72 (11.35)		
	≥5	91.8 (12.28)		

Dependent child	Has	86.57 (13.67)	2.791	0.097
	None	78.81 (22.92)		

A person who usually cares and helps	Marriage partner	87.69 (14.84)	0.603	0.905
	Children	84.65 (13.70)		
	Neighbors and others	85.63 (16.8)		

Meeting	Senior citizen's center	88.04 (11.72)	2.619	0.041
	Senior college	88.33 (21.65)		
	Senior volunteer group	101.00 (6.08)		
	None	82.40 (14.59)		

Number of meetings	Once a week	90.97 (15.45)	3.764	0.003
	Once in two weeks	80.85 (10.25)		
	Once a month	86.64 (10.95)		
	Once in two months	81.71 (14.38)		

Occupation status	Has	88.46 (15.09)	0.527	0.469
	None	85.49 (14.78)		

Economic level	Low	97.55 (13.16)	10.201	0.001
	Medium	85.32 (13.28)		
	High	77.55 (16.10)		

Monthly allowance	≥100,000 won	82.04 (14.48)	1.708	0.033
	≥200,000 won	87.08 (9.85)		
	≥300,000 won	83.12 (14.14)		
	≥400,000 won	86.66 (16.06)		
	≥500,000 won	91.13 (15.89)		

Subjective health status	Very healthy	65.00 (12.44)	9.556	0.001
	Healthy	82.60 (13.55)		
	Average	84.53 (14.24)		
	Unhealthy	91.46 (9.85)		
	Very unhealthy	110.80 (9.73)		

Disease status	Has	84.82 (13.51)	1.233	0.269
	None	88.02 (17.13)		

**Table 8:** Correlation between depression level, quality of sleep, and quality of life.

Domain	Physical domain	Psychological domain	Social domain	Living environment domain
Depression	0.177 (0.054)	0.270 (0.003)	0.245 (0.007)	−0.205 (0.024)
Quality of sleep	−0.089 (0.311)	−0.455 (0.001)	−0.075 (0.365)	0.419 (0.001)

**Table 9:** Factors affecting the quality of life.

Variable	Physical domain		Psychological domain		Social domain		Living environment domain	
	*β*	*p*	*β*	*p*	*β*	*p*	*β*	*p*
Constant		0.610		0.333		0.478		0.983
Gender	0.089	0.478	0.166	0.123	0.016	0.886	0.104	0.363
Age (year)	−0.064	0.635	0.020	0.865	−0.019	0.875	0.050	0.687
Religion	−0.011	0.911	0.164	0.058	0.065	0.477	0.112	0.222
Education	0.164	0.171	−0.144	0.159	−0.139	0.200	−0.043	0.693
Marital status	−0.167	0.336	0.090	0.545	−0.038	0.811	−0.052	0.741
Living together	0.008	0.961	−0.003	0.985	−0.010	0.947	0.016	0.918
Number of children	0.302	0.010	−0.057	0.568	0.049	0.639	0.031	0.770
Dependent child	0.010	0.919	−0.142	0.099	−0.009	0.919	−0.083	0.366
A person who usually cares and helps	0.028	0.800	−0.180	0.056	0.098	0.322	−0.075	0.453
Meeting	−0.051	0.770	0.015	0.918	0.194	0.223	0.148	0.354
Number of meetings	−0.069	0.693	−0.095	0.523	−0.232	0.143	−0.107	0.501
Occupation status	0.048	0.649	−0.287	0.002	0.109	0.255	−0.041	0.673
Economic level	0.090	0.407	0.024	0.801	−0.288	0.004	−0.027	0.783
Monthly allowance	0.044	0.671	−0.038	0.668	0.092	0.336	−0.171	0.077
Subjective health status	0.071	0.582	−0.018	0.869	0.280	0.018	−0.070	0.555
Disease status	−0.140	0.179	0.016	0.858	0.021	0.822	−0.216	0.025
Depression	0.107	0.318	0.145	0.117	0.121	0.215	−0.049	0.616
Quality of life	−0.015	0.890	−0.348	0.001	0.158	0.102	0.436	0.001

## Data Availability

The data used to support the findings of this study are available from the corresponding author upon request.
